This article has been retracted.

# Prognostic Value of Immunotyping Combined with Targeted Therapy in Patients with Non-Small-Cell Lung Cancer and Establishment of Nomogram Model

**DOI:** 10.1155/2022/3049619

**Published:** 2022-05-14

**Authors:** Sha Tian, Yinmei Guo, Jiajun Fu, Zijing Li, Jing Li, Xuefei Tian

**Affiliations:** ^1^Department of Internal Medicine, College of Integrated Chinese and Western Medicine, Hunan University of Chinese Medicine, China; ^2^Hunan Key Laboratory of Traditional Chinese Medicine Prescription and Syndromes Translational Medicine, Hunan University of Chinese Medicine, China; ^3^Medical School, Hunan University of Chinese Medicine, China; ^4^Acupuncture-Moxibustion-Tuina and Rehabilitation, Hunan University of Chinese Medicine, China; ^5^Department of Oncology, The First Hospital of Hunan University of Chinese Medicine, China

## Abstract

**Objective:**

Bioinformatics methods were used to analyze non-small-cell lung cancer gene chip data, screen differentially expressed genes (DEGs), explore biomarkers related to NSCLC prognosis, provide new targets for the treatment of NSCLC, and build immunotyping and line-map model.

**Methods:**

NSCLC-related gene chip data were downloaded from the GEO database, and the common DEGs of the two datasets were screened by using the GEO2R tool and FunRich 3.1.3 software. DAVID database was used for GO analysis and KEGG analysis of DEGs, and protein-protein interaction (PPI) network was constructed by STRING database and Cytoscape 3.8.0 software, and the top 20 hub genes were analyzed and screened out. The expression of pivot genes and their relationship with prognosis were verified by multiple external databases.

**Results:**

159 common DEGs were screened from the two datasets. PPI network was constructed and analyzed, and the genes with the top 20 connectivity were selected as the pivotal genes of this study. The results of survival analysis and the patients' survival curve was reflected in the line graph model of NSCLC.

**Conclusion:**

Through the screening and identification of the VIM-AS1 gene, as well as the analysis of immune infiltration and immune typing, the successful establishment of the rosette model has a certain guiding value for the molecular targeted therapy of patients with non-small-cell lung cancer.

## 1. Introduction

Lung cancer has become the main cause of cancer death worldwide, and its incidence and mortality rate has increased significantly in recent years [1]. A series of studies have shown that smoking, air pollution, occupational exposure, and other factors are related to the occurrence of lung cancer [2]. Among all patients with lung cancer, non-small-cell lung cancer (NSCLC) accounts for about 85%. Patients with early NSCLC have an acceptable prognosis after surgical treatment [3]. In recent years, although great progress has been made in the early diagnosis and treatment of NSCLC, its prognosis is still not optimistic. Therefore, it is important to find biomarkers that can accurately predict patient outcomes. With the development of science and technology, the establishment of a large number of genomic microarray databases provided an important basis for studying the differentially expressed genes (DEGs) in lung cancer [4].

The incidence and mortality of lung cancer showed an obvious upward trend [5]. The treatment of lung cancer has developed from traditional hand surgery, radiotherapy, and chemotherapy to comprehensive treatment including molecular targeting and immunotherapy. The classification of lung cancer has also been further subdivided into molecular subtypes based on driver genes, and NSCLC has entered an era of accurate diagnosis and treatment [6]. Therefore, it is important to further study the diagnostic markers and therapeutic targets with high specificity for lung cancer. There are a lot of sequencing data in the GEO database, and the bioinformatics method is used to mine genes with research value, which provides a direction for further in-depth research [7–10].

In this study, two lung cancer gene expression profiles GSE19804 and GSE335332 were selected from the GEO database to screen out DEGs and explore their functions in the occurrence and development of NSCLC. It has a certain guiding significance for the establishment of the immunoassay and puncture angiography model.

## 2. Materials and Methods

### 2.1. Chip Data Extraction

Among them, the GSE19804 dataset was published with 60 NSCLC samples and 60 normal lung tissue samples collected. The GSE33532 dataset was published, and 80 NSCLC samples and 20 normal lung tissue samples were collected. In addition, we have used the ComBat algorithm to remove the identified batch effects of GSE19804 and GSE33532 in this study.

### 2.2. Screening of Differential Genes between NSCLC and Normal Lung Tissue

Using the default Benjamini and Hochberg false discovery rate methods, the *P* values were adjusted to reduce the false-positive rate. Using adjusted *P* < 0.05, ∣log2FC | >2 as the cutoff criteria, Fun-Rich3.1.3 was used for the two datasets. The DEGs took the intersection and finally selected the common DEGs.

### 2.3. Enrichment Analysis of the Differential Genes

GO and KEGG analysis of DEGs, and visualization of functional analysis (cell components, molecular functions, biological processes, and signaling pathways) of coexpressed DEGs.

### 2.4. Construction of the PPI Network and the Screening of the Hub Genes

In the analysis of plasma-albumin interactions, PPI analysis of DEGs was performed with the reliabilityscore ≥ 0.4and the maximum interactionnumber = 0as the boundary value. Subsequently, the cytoHubba plug-in in Cytoscape3.8.0 (http://www.cytoscape.org/) was used. The top 20 with high degree of connectivity with surrounding genes were screened. Two genes act as hinge genes. cytoHubba uses several topological algorithms to predict and explore the interrelation systems between important nodes and subnetworks in a given network. In network extension theory, the connect degree (*K*) is defined as the number of connections between a node and other nodes in the network, that is, the number of adjacent proteins.

### 2.5. Survival Analysis

The 20 hub genes with overall survival (*P* < 0.05) (NSCLC) were selected, and survival curves were plotted by the Kaplan-Meier method.

### 2.6. Statistical Analysis

The data were expressed as mean ± SD (standard deviation). We evaluated the continuous data between the two groups using the *t*-test. In addition, statistical analysis was performed using GraphPad Prism 8 and R software (Version 3.6.1), and the difference of *P* < 0.05 was considered statistically significant.

## 3. Result

### 3.1. Screening of Differentially Expressed Genes of lncRNA

We from the UCSC XENA (https://xenabrowser.net/datapages/) download through Toil process unified processing TCGA and GTEx TPM RNAseq data format. The figure shows the comparison of the expression of VIM-AS1. Finally, it was concluded that VIM-AS1 was significantly expressed in bladder urothelial carcinoma BLCA, breast invasive carcinoma BRCA, hepatocellular carcinoma LIHC, lung adenocarcinoma LUAD, lung squamous cell carcinoma LUSC, skin melanoma SKCM, gastric cancer STAD, and thyroid cancer THCA, with statistically significant results (*P* < 0.05) (Figure 1).

### 3.2. lncRNA Coexpressed Genes

According to the expression of VIM-AS1 in TCGA lung adenocarcinoma LUAD, | logFC | >1 and padj < 0.05 the difference of molecular has 6122. And padj | logFC | >1.5 <0.05 the difference of molecular has 3348; 2 and padj | logFC | > <0.05 the difference of molecular has 1922(Table 1).

### 3.3. Volcanic Map and Heat Map Analysis

The volcano map is used to show the results of the different analyses. There were 763 molecules with logFC > 2 and PADJ < 0.05. There were 1159 different molecules with logFC < −2 and PADJ < 0.05 (Figure 2). In the TCGA lung adenocarcinoma, LUAD VIM-AS1 is divided into the high expression and low expression in the two groups after the present common gene expression differences, and high VIM-AS1 gene expression related genes CCDC37, ZMYND10, TTC16, DLEC1, and TTLL9; genes associated with low expression of VIM-AS1 include S100P, INSL4, GPX2, F2, and CA12 (Figure 3).

### 3.4. GO and KEGG Functional Enrichment Analyses

We used the clusterProfiler package to analyze the gene ontology (GO) enrichment analysis of the input gene list, including biological processes (BP), cellular components (CC), and molecular function (MF), and KEGG pathway enrichment analysis (Figure 4(a)). As can be seen from the figure, GO functional enrichment pathways are mainly concentrated in cilium movement pathway (GO: 0003341), microtubule bundle formation pathway (GO: 0001578), and axoneme assembly pathway (GO: 0035082). Reference gene set H.all.v7.0.symbols. In the GMT [Hallmarks], the selected visual dataset is HALLMARK_G2M_CHECKPOINT withNES = −2.319,padj = 0.007, andFDR = 0.003, and the results indicate that this dataset is significantly enriched in blue on the right (ViM-AS1 low expression group), and VIM-AS1 may be associated with this dataset. It can be seen from the figure that the enrichment pathways of KEGG are neuroactive ligand-receptor interaction (HSA04080), metabolism of xenobiotics by cytochrome (HSA00980), and other pathways (Figure 4(b)).

### 3.5. Analysis of Immune Infiltration and Immune Typing

Marker genes of 24 kinds of immune cells were extracted from the Immunity official website database, and the infiltration of 24 kinds of immune cells in lung adenocarcinoma LUAD was analyzed by ssGSEA method, and the correlation between VIM-AS1 and these 24 kinds of cells was analyzed by Spearman's correlation method. The Wilcoxon rank-sum test was used to analyze the difference in NK cell, Th1 cell, and Th2 cell infiltration levels between the high and low expression groups of VIM-AS1 (Figure 5).

### 3.6. Correlation Analysis of Basic Clinical Features

The Kruskal-Wallis rank-sum test was used to compare the relationship between the expression of VIM-AS1 and a series of basic clinical characteristics of TCGA lung adenocarcinoma LUAD. There were significant differences in the T and N stages of TCGA lung adenocarcinoma and gender (*P* < 0.001), but there were no significant differences in M stage, age, smoking status, TP53 status, and KRAS status, and the relevant data were not statistically significant (*P* > 0.05) (Figure 6). Moreover, the statistical difference of VIM-AS1 gene expression only exists between stage I and stage IV (Figure 6(a)) as well as PD and CR (Figure 6(d)). Other progression period comparisons were not found with statistical significance (*P* > 0.05).

### 3.7. KM Plot Curve Analysis

The figure shows the Kaplan-Meier plot drawn by the survMiner package to evaluate the prognostic value of VIM-AS1 in the overall survival of lung adenocarcinoma. The gene expression values were divided into high and low expression groups according to the median. Low expression of VIM-AS1 was associated with poorer. Low expression of VIM-AS1 was associated with poorer disease-specific survival (HR = 0.47 (0.32-0.69), *P* < 0.001). The risk table in the lower part records the number of people who are still being followed up at each time point (Figure 7).

### 3.8. Nomogram Analysis

Figure 8 is a nomogram showing the prognostic prediction model, including primary therapy outcome, pathologic stage, and VIM-AS1, with a C-index of 0.736 (0.725-0.791). The value of the C-index is generally between 0.5 and 1 (Figure 8). The training set was used to determine the test set and its C-index, respectively. The value range of the model is [3, 10, 30, 40, 50] for the random forest and [100, 300, 500, 600] for CatBoost. Default values were set for other parameters in the machine learning algorithms.

## 4. Discussion

Lung cancer is now the leading cause of cancer-related death worldwide. However, since most NSCLC patients are already in an advanced stage when diagnosed and have no chance of surgery, the 5-year survival rate is only 16% [11]. The complex biological behavior of lung cancer tissue involves many genes and related pathways, and the mechanism of its occurrence and development is not very clear at present [12–16]. This study was aimed at screening out differential genes and then exploring biomarkers related to NSCLC prognosis, to provide new ideas for diagnosis and treatment of NSCLC [17–19].

In this study, 159 DEGs between NSCLC and normal lung tissue were screened by mining two gene cores GSE19804 and GSE33532. Through STRING and Cytoscape3.8.0, the PPI network of DEGs was constructed and calculated, and 20 pivot genes were finally determined [20–25]. However, adverse drug reactions and drug resistance limit the ultimate effect of chemotherapy. New strategies to complement conventional chemotherapy are therefore urgently needed [26–29].

Systemic chemotherapy has always been the main treatment option for these patients. At the beginning of the 21st century, with the deepening of molecular biology research, NSCLC can be classified into molecular phenotypes according to the different expressions of various molecular markers, and new drugs can be developed to carry out targeted individual molecular targeted therapy by targeting the driving genes related to tumor genesis and development [30–34]. At present, personalized therapy based on molecular markers has moved from the laboratory to the clinic [35]. In this study, we found that the expression of VIM-AS1 is significantly higher in NSCLC tissues than that in adjacent normal tissues, and VIM-AS1 expression is positively correlated with tumor pathological grades, TNM stages, and distant metastasis of NSCLC, as well as the clinical outcomes of NSCLC patients. VIM-AS1 may exert an oncogenic role in the NSCLC cells through epigenetic suppression of p21 expression and serve as a novel prognostic biomarker in human NSCLC.

In conclusion, through screening and identification of genes for survival and prognosis of lung adenocarcinoma, as well as analysis of immune infiltration and immune typing, the successful construction of the line graph model has a certain guiding value for the molecular targeted therapy. VIM-AS1 gene may be a biomarker to evaluate the prognosis of NSCLC patients, providing a new idea for the diagnosis and treatment of NSCLC.

## Figures and Tables

**Figure 1:** lncRNA VIM-AS1 gene expression difference (NS, *P* ≥ 0.05; ∗, *P* < 0.05; ∗∗, *P* < 0.01; ∗∗∗, *P* < 0.001).

**Figure 2:** Volcano diagram of differential expression of lncRNA.

**Figure 3:** VIM-AS1 was divided into heat maps of coexpressed differentially expressed genes with high and low expression.

**Figure 4:** (a and b) Visualization of enrichment analysis results—bubble chart.

**Figure 5:** Spearman's correlation method was used to analyze the correlation between VIM-AS1 and 24 kinds of cells.

**Figure 6:** (a–i) Clinical correlation analysis.

**Figure 7:** (a–c) The Kaplan and Meier curves.

**Figure 8:** Nomogram analysis.

**Table 1:** Differentially expressed genes in HTSEQ-count data of VIM-AS1.

Gene_id	log2FoldChange	*P* value	gene_name	gene_biotype	cor_pvalue	Correlation
ENSG00000198804	-0.36801791	3.71E-02	MT-CO1	protein_coding	1.43E-01	0.0648168
ENSG00000168878	0.52560666	1.95E-01	SFTPB	protein_coding	3.44E-03	0.129034156
ENSG00000198886	-0.58391127	1.60E-03	MT-ND4	protein_coding	4.00E-01	-0.037196438
ENSG00000210082	-0.532619	5.19E-03	MT-RNR2	Mt_rRNA	2.46E-01	-0.051260432
ENSG00000198938	-0.28263912	1.29E-01	MT-CO3	protein_coding	7.07E-03	0.118858014
ENSG00000075624	-0.05543028	5.96E-01	ACTB	protein_coding	5.43E-04	0.152344194
ENSG00000211896	0.12159637	7.11E-01	IGHG1	IG_C_gene	8.02E-01	-0.011086863
ENSG00000198712	-0.55702706	2.35E-03	MT-CO2	protein_coding	7.42E-01	-0.014558908
ENSG00000156508	-0.18184162	2.48E-01	EEF1A1	protein_coding	3.96E-01	0.037512426
ENSG00000087086	-0.81424428	4.13E-05	FTL	protein_coding	1.51E-02	-0.107224416
ENSG00000185303	2.36713141	3.47E-07	SFTPA2	protein_coding	1.23E-07	0.231550575
ENSG00000198727	-0.25538089	1.77E-01	MT-CYB	protein_coding	2.24E-02	0.100861282
ENSG00000198763	-0.62633062	1.94E-03	MT-ND2	protein_coding	9.94E-01	-0.00031901
ENSG00000184009	-0.25108983	3.03E-02	ACTG1	protein_coding	5.43E-01	-0.026912478

## Data Availability

The data used to support this study are available from the corresponding author upon request.
